The article "Molecular Diversity of Legume Root-Nodule Bacteria in Kakadu National Park, Northern Territory, Australia" was published in 2007. Journal: PLoS One.

# Molecular Diversity of Legume Root-Nodule Bacteria in Kakadu National Park, Northern Territory, Australia

**DOI:** 10.1371/journal.pone.0000277

**Published:** 2007-03-07

**Authors:** Bénédicte Lafay, Jeremy J. Burdon

**Affiliations:** Commonwealth Scientific and Industrial Research Organisation (CSIRO) Plant Industry, Centre for Plant Biodiversity Research, Canberra, Australia; The Institute for Genomic Research, United States of America

## Abstract

**Background:**

Symbiotic relationships between leguminous plants (family Fabaceae) and nodule-forming bacteria in Australia native ecosystems remain poorly characterized despite their importance. Most studies have focused on temperate parts of the country, where the use of molecular approaches have already revealed the presence of *Bradyrhizobium, Ensifer* (formerly *Sinorhizobium*), *Mesorhizobium* and *Rhizobium* genera of legume root-nodule bacteria. We here provide the first molecular characterization of nodulating bacteria from tropical Australia.

**Methodology/Principal Findings:**

45 nodule-forming bacterial strains, isolated from eight native legume hosts at eight locations in Kakadu National Park, Northern Territory, Australia, were examined for their genetic diversity and phylogenetic position. Using SSU rDNA PCR-RFLPs and phylogenetic analyses, our survey identified nine genospecies, two of which, *Bradyrhizobium* genospp. B and P, had been previously identified in south-eastern Australia and one, *Mesorhizobium* genospecies AA, in southern France. Three of the five newly characterized *Bradyrhizobium* genospecies were more closely related to *B. japonicum* USDA110, whereas the other two belonged to the *B. elkanii* group. All five were each more closely related to strains sampled in various tropical areas outside Australia than to strains known to occur in Australia. We also characterized an entirely novel nodule-forming lineage, phylogenetically distant from any previously described rhizobial and non-rhizobial legume-nodulating lineage within the Rhizobiales.

**Conclusions/Significance:**

Overall, the present results support the hypothesis of tropical areas being centres of biodiversity and diversification for legume root-nodule bacteria and confirm the widespread occurrence of *Bradyrhizobium* genosp. B in continental Australia.

## Introduction

Members of the family Fabaceae represent about 10% of the estimated 18,000 native plant species in Australia where they occur in nearly all vegetation types [1]. Their ecological success may reflect the advantage that legumes gain in soils of low fertility (a characteristic of the majority of Australian ecosystems) by associating with nitrogen-fixing bacteria. Indeed, relationships between leguminous plants and their nitrogen-fixing bacterial symbionts were shown to be of particular significance for reforestation and native ecosystem restoration in Australia's low fertility soils [2], [3], [4]. However, the study of diversity among the symbiotic microbiota of Australian native legumes is poorly advanced as most assessments have relied on growth characteristics and nodulation experiments which only separate nodulating bacteria into fast-versus slow-growers, and according to their nitrogen-fixing efficiency [5], [6], [7], [8], [9].

The article "Molecular Diversity of Legume Root-Nodule Bacteria in Kakadu National Park, Northern Territory, Australia" was published in 2007. Journal: PLoS One.

The legume root-nodule bacteria are collectively known as ‘rhizobia’ and belong to one of the six genera [10], *Rhizobium, Mesorhizobium, Ensifer* (formerly *Sinorhizobium*), *Allorhizobium, Bradyrhizobium, Azorhizobium* [11]. Molecular data have shown that these bacteria actually constitute a polyphyletic assemblage of alphaproteobacteria, which form the Rhizobiales group with recently identified non-rhizobia nodulating taxa [12], [13], [14], [15], [16], [17] and a number of non-nodulating lineages. These latter include plant or animal pathogens, epiphytes, animal symbionts, or free-living bacteria. Additionally, bacteria capable of symbiotically associating with legumes have been identified among betaproteobacteria [18], [19], [20] and possibly gammaproteobacteria [21].

The few studies that have applied molecular techniques to the characterization of Australian nodulating bacteria confirmed that both fast-and slow-growing rhizobia occur naturally and detected three of the six rhizobia genera [13], [22], [23], [24] among the isolates tested. A number of *Bradyrhizobium, Mesorhizobium* and *Rhizobium* genospecies were identified on the basis of SSU-rDNA sequence data. None of these corresponded to previously described species [22], [23]. In general, *Bradyrhizobium* species predominated among rhizobia isolated from a diverse range of native legume hosts sampled from sites across southern Australia [13], [22], [23], [24]. The various genospecies (i.e., species characterized at the genomic level only) exhibited different distribution patterns. For example, of the two most abundant genospecies that were identified in the Australian Capital Territory (ACT) and New South Wales (NSW), genospecies B occurred in a range of different climatic and edaphic conditions across the whole continent whereas genospecies A was restricted to more temperate regions [22], [23].

To further knowledge of Australian rhizobial diversity and ecology in the context of re-establishment of vegetation in nitrogen-deficient soils, we conducted a preliminary survey aiming at characterizing nodulating bacteria derived from the northern tropical part of Australia.

The article "Molecular Diversity of Legume Root-Nodule Bacteria in Kakadu National Park, Northern Territory, Australia" was published in 2007. Journal: PLoS One.

## Results

### Phylogenetic Diversity of Northern Territory Legume Root-Nodule Bacteria

Forty-five isolates collected in Kakadu National Park, Northern Territory, Australia were characterized by SSU rDNA PCR-RFLPs (Table 1). Nine different Rhizobiales genospecies were detected. None corresponded to described species and only three to previously characterized genospecies. These latter were *Bradyrhizobium* genospp. B and P, that have been identified among south-eastern Australia rhizobial communities [22] and isolated from various legume hosts from south Queensland to Tasmania [22], [23], and *Mesorhizobium* genosp. AA, that we identified among the nodule isolates sampled from *Cytisus scoparius* in the South of France [13]. The six yet uncharacterized genospecies that we identified were arbitrarily named V, W, X, Y, Z, and AL so as to complement the denominations applied in our earlier studies of rhizobia communities [13], [22]. Genospecies V to Z, were members of the genus *Bradyrhizobium* whereas genospecies AL showed no strong SSU rDNA sequence similarity to any of the 8 nodulating lineages within the Rhizobiales [11], [13], [14]. The *Bradyrhizobium* genospecies could be divided into two groups on the SSU rDNA basis. Genospecies V, W, and X SSU rDNA sequences were *B. japonicum*-like whereas Y and Z sequences were more similar to *B. elkanii* lineage sequences. Indeed, *Bradyrhizobium* taxa in that latter group possess SSU rDNAs which appear to have evolved from a recombination event between ‘typical’ *Bradyrhizobium* and *Mesorhizobium* SSU rDNAs [22], [25]. Since this can result in spurious branching, we ran separate phylogenetic analyses. Genospecies V, W, and X grouped with *Bradyrhizobium japonicum* USDA110 and genospecies V and X formed a separate lineage with *Bradyrhizobium* sp. phym 6a and *Bradyrhizobium* sp. ORS 3259 (Figure 1A). Genospecies Y and Z formed a separate cluster (internal branch length statistically different from zero), although only poorly supported by 100 bootstrap replicates (<50%) within the *B. elkanii* lineage (Figure 1B). Interestingly, irrespective of their clustering with *B. japonicum* or *B. elkanii*, all the *Bradyrhizobium* genospecies characterized during this survey had closest phylogenetic relatives isolated from diverse legume hosts outside Australia that are all tropical or subtropical in origin (Genospecies V, W and X: Barro Colorado Island, Panama (AY528712), Costa Rica (AF514704), Senegal (AF514798, AY039015), Thailand (AB072419, AB07420), and Hubei, China (AF530465); Genospecies Y and Z: Costa Rica (AF514703) and Barro Colorado Island, Panama (AY187548)). The phylogeny reconstruction confirmed that genospecies AL was different from any previously reported nodulating member of the Rhizobiales. The most closely related nodulating taxon is *Methylobacterium nodulans* although other non-nodulating taxa among the Rhizobiales are more closely related (Figure 1C).

The article "Molecular Diversity of Legume Root-Nodule Bacteria in Kakadu National Park, Northern Territory, Australia" was published in 2007. Journal: PLoS One.

**Figure 1:** Phylogenetic relationships of the six newly characterized Rhizobiales genospecies. Internal branches with length not significantly different from zero are shown as a dashed line. Numbers correspond to percentage bootstrap support for internal branches based on 100 replications (only values above 50% are shown). Scale bar corresponds to numbers of nucleotide substitution per site. A) Phylogenetic position of genospecies V,W and X within the *B. japonicum* group. B) Phylogenetic position of genospecies Y and Z within the *B. elkanii* group. C) Phylogenetic position of genospecies AL within Rhizobiales.

**Table 1:** Distribution of the nodulating taxa, identity and numbers of isolates according to site of origin and legume host^a^

Sampling sites^b^	Caesalpinioideae		Mimosoideae		Papilionoideae			
	*Cm*	*So*	*Cu*	*Ng*	*Ic*	*Ih*	*Il*	*Is*
South Alligator (13°29′S/132°22′E) rainforest, loam flat, undisturbed			P(1)					
Spring Peak Range (12°58′S/132°27′E) woodland, rocky hill, undisturbed	B(2) W(3)							
Coronation Hill (13°35′S/132°36′E) woodland, schist hill, disturbed		P(1) Z(1)			B(3) AA(1)	B(4) X(1) AA(2)		
Fisher airstrip (13°33′S/132°38′E) woodland, loam flat, disturbed				B(4)			B(7)	
Alligator River between Parks H.Q. & Jabiru Drive (12°42′S/132°38′E) woodland, loam flat, undisturbed					B(3)			B(1)
Jabiru Drive opposite Crocodile Hotel (12° 40′ S/132° 49′ E) woodland, rocky loam, disturbed							B(4)	
Jabiluka (12°29′S/132°53′E) woodland, sandy hill, undisturbed	V(1)							
Mount Cahill base (12°52′S/134°42′E) woodland, sandy loam slope, undisturbed							Y(1) AL(1)	
Mount Cahill top (near look-out) (12°52′S/134°42′E) woodland, rocky hill, disturbed	B(1)						B(2) Z(1)	

a Cm, Chamaecrista mimosoides; So, Senna obtusifolia; Cu, Cathormion umbellatum; Ng, Neptunia gracilis; Ic, Indigofera colutea; Ih, Indigofera hirsuta; Il, Indigofera linifolia; Is, Indigofera saxicola.

b Latitude/longitude, vegetation, soil and disturbance conditions are given for each site.

### Geographical and Host Distribution

The incidence of the nine legume-nodulating taxa among the total isolate sample was highly imbalanced (Table 1). One genospecies constituted the bulk of the 45 strains (69%) whereas the other eight were each present 1–3 times only. *Bradyrhizobium* genosp. B, the most abundant (31 strains out of 45), was isolated from six different hosts, covering all three sub-families of the Fabaceae. *Bradyrhizobium* genosp. P was not recovered from any of these six hosts but occurred on the other two, *Senna obtusifolia* (Caesalpinioideae) and *Cathormion umbellatum* (Mimosoideae), from which genospecies B was not isolated. Genospecies P was only isolated once on each host but the total number of strains for each host species was also very small (two and one respectively). Each of the six newly characterized genospecies V, W, X, Y, Z, and AL as well as genospecies AA were isolated from legume host(s) also associated with *Bradyrhizobium* genosp. B. Additionally, *Bradyrhizobium* genosp. Z was isolated from *Senna obtusifolia* from which *Bradyrhizobium* genosp. B was not recovered. Genospecies Z and AA represented by two and three strains respectively were isolated from two hosts. The two *Bradyrhizobium* genosp. Z strains originated from different sites (Coronation Hill for *Senna obtusifolia* and Jabiru Drive for *Indigofera linifolia*) whilst *Mesorhizobium* genosp. AA nodulated two *Indigofera* species, *I. colutea* (one strain) and *I. hirsuta* (two strains), at the same site (Coronation Hill). In contrast, all three strains of *Bradyrhizobium* genosp. W were detected on just one host, *Chamaecrista mimosoides* (Caesalpinioideae), at Spring Peak Range.

The article "Molecular Diversity of Legume Root-Nodule Bacteria in Kakadu National Park, Northern Territory, Australia" was published in 2007. Journal: PLoS One.

The sites sampled represented various soil, vegetation and disturbance conditions (Table 1). No link between these respective characteristics and the nature of the genospecies identified at a given site was apparent. However, this could not be assessed statistically because of the sparse data. *Bradyrhizobium* genosp. B was found to occur at all but two sites. For these latter, only one isolate was available. Importantly, most of the genospecies characterized in the course of this study occurred at undisturbed sites. A notable exception was *Mesorhizobium* genosp. AA.

## Discussion

The identity and community structure of legume root-nodule bacteria in tropical Australia has been addressed by a few studies that assessed bacterial growth rate, nodulation ability and/or the nitrogen fixation efficiency of *Acacia* spp. at Groote Eylandt, Northern Territory [7], [26] and of *Acacia* spp. [9], [27] and various legumes in Queensland [28], [29], [30], [31]. These studies concluded that legume root-nodule bacteria in northern Australia were slow-growers (‘cowpea cross-inoculation group’) [31], [32], with 100 strains isolated from *Acacia mangium* in North Queensland all being shown to be *Bradyrhizobium* spp. [27]. More recently, this claim has gained some support from molecular evidence. SSU-rDNA comparison demonstrated that all strains isolated from *Acacia* spp. in sub-tropical south Queensland were indeed *Bradyrhizobium* spp. [23]. In contrast, *Rhizobium tropici* (genospecies Q) could be identified among strains isolated from *Acacia* spp. in more southern temperate regions, and more importantly from *Acacia melanoxylon* which was also present at one of the Queensland sampling sites [23].

The article "Molecular Diversity of Legume Root-Nodule Bacteria in Kakadu National Park, Northern Territory, Australia" was published in 2007. Journal: PLoS One.

Our present results extend this work to assess genetic relatedness among legume root-nodulating strains collected from Kakadu National Park in Northern Australia. Of the 45 strains that we characterized using the same methodological approach applied in our earlier analyses of southern Australian legume root-nodulating communities, most (91%) were indeed *Bradyrhizobium* species. It thus appears, in agreement with earlier studies in south-eastern Australia [5], [6], [8], [9], [22], [23], Queensland [23], [27], [28], [29], [30], [31] and Western Australia [24], [33], that *Bradyrhizobium* is by far the most common lineage present among legume root-nodule bacteria throughout Australia. Interestingly, *Bradyrhizobium* genosp. B was predominant in the Northern Territory, thus lending support to the hypothesis that it is the most widespread genospecies occurring in Australia [23]. As previously observed, it was found to be promiscuous, and exhibited a broad host range encompassing all three Fabaceae subfamilies. However, as we observed in south-eastern Australia [22], [23], a small number of strains (four) did not belong to that lineage. In this regard, the diversity of legume root-nodule bacteria in tropical Australia appears to be little different from that found in tropical areas of other parts of the world [14], [34], [35], [36].

Nine genospecies were identified among 45 strains collected over a small area (Kakadu National Park) whereas only 21 genospecies were detected among 745 strains collected in ACT and NSW [23]. Nine of the latter genospecies were also identified among 118 isolates collected over a wider area of south-eastern Australia including southern Queensland and Tasmania [23]. However, seven out of the nine genospecies occurring in the Northern Territory had not been previously found among the 863 (745+118) isolates from south-eastern Australia. Nor did they correspond to any of the genospecies characterized by partial SSU rDNAs in Western Australia [24]. Furthermore, we detected a novel strain that was not related to any of the currently described legume root-nodule alpha-and beta-proteobacterial lineages [11], [13], [14]. Indeed, genospecies AL clearly stands apart from genera where nodulating taxa have been identified and cannot be ascribed to any of the current, formally described lineages. It thus represents an entirely novel lineage capable of associating symbiotically with legumes and is probably a new genus within the Rhizobiales. Our results thus provide some support for the claims that tropical regions are one of the main areas of legume biodiversity [37] and that tropical forests are centres of origin of legume root-nodule bacteria [32], [38].

The article "Molecular Diversity of Legume Root-Nodule Bacteria in Kakadu National Park, Northern Territory, Australia" was published in 2007. Journal: PLoS One.

However, of the four non-*Bradyrhizobium* isolates, three corresponded to *Mesorhizobium* genosp. AA which had previously been identified on another continent [13]. Accordingly, within the *Mesorhizobium huakuii* phylogenetic cluster, in contrast to two (T and U) of the three *Mesorhizobium* genospecies that were found in south-eastern Australia [22], genospecies AA is more closely related to other lineages identified in other parts of the world [13]. There is a possibility that exotic rhizobia were introduced with planting stock used to revegetate mine site areas of Kakadu National Park [3]. The occurrence of *Mesorhizobium* genosp. AA isolates at the Coronation Hill mine site in Kakadu National Park may thus result from the site disturbance.

Restoration of land plant communities and land rehabilitation involving leguminous plants require that appropriate rhizobial symbionts are present in the often degraded soils. Our preliminary survey shows that, although some genospecies had previously been identified in temperate Australia, the nodulating bacteria in tropical Australia are overall more diverse than those found in other part of the continent and that some genospecies may be typically tropical in origin. This should thus be taken into account when planning re-vegetation programmes.

## Materials and Methods

### Bacterial Strains

The 45 isolates used in this study were provided by the Alligator Rivers Regional Institute (ARRI) and Environmental Research Institute of the Supervising Scientist (ERISS), Kakadu National Park, Australia. These nodulating bacteria had been collected and authenticated in 1991 and 1992 from 8 legume species representing 5 genera belonging to the Caesalpinioideae, Mimosoideae and Papilionoideae at 8 locations in Kakadu National Park, Northern Territory, Australia (Table 1) [39].

### DNA Preparation

Bacterial DNA was prepared using the method of Sritharan and Barker [40]. Bacteria were grown on yeast extract mannitol agar (YMA) medium at 28°C [41] for three to ten days depending on the strain and species until colonies appear. Single colonies were picked and suspended in 100 µl of 10 mM Tris pH 8.0, 1 mM EDTA, 1% Triton X-100 solution and boiled for 5 min. After a single chloroform extraction, 5 µl of the supernatant were used in the amplification reaction.

The article "Molecular Diversity of Legume Root-Nodule Bacteria in Kakadu National Park, Northern Territory, Australia" was published in 2007. Journal: PLoS One.

### SSU rRNA Gene Amplification

Primers corresponding to positions 8 to 28 and 1492 to 1509 [42] in the *Escherichia coli* SSU rRNA sequence (J01695) were used for amplification of the SSU rRNA genes by polymerase chain reaction. PCR reactions were carried out in a 100 µl volume containing 5 µl of template DNA solution, 50 pmol of each of the two primers, 200 µM dNTP and 2.5 U of Amplitaq DNA polymerase (Perkin Elmer) in Amplitaq DNA polymerase reaction buffer (10 mM Tris-HCl pH 8.3, 50 mM KCl, 1.5 mM MgCl_2_). Amplifications were performed using the following temperature profile: an initial cycle consisting of a denaturation step at 95°C for 5 min, an annealing step at 52°C for 120 sec and an extension step at 72°C for 90 sec; then 30 cycles of denaturation at 94°C for 30 sec, annealing at 52°C for 60 sec, and extension at 72°C for 60 sec; and a final extension step at 72°C for 5 min.

### SSU rDNA PCR-RFLPs

Aliquots (10 µl) of PCR products were digested with restriction endonucleases [43]. A combination of four enzymes (*Hha*I, *Hin*fI, *Msp*I, *Rsa*I), which distinguished rhizobial species [43] was used. Restricted fragments were separated by electrophoresis on 3% NuSieve 3:1 agarose gels at 80V for 5 h, and visualized by ethidium bromide staining.

### PCR Product Sequencing

Representative examples of isolates possessing a PCR-RFLP genotype distinct from those that we previously identified [13], [22], [23] were used in a subsequent sequence comparison. Small-subunit rDNA PCR products were purified using a Wizzard™ PCR Preps DNA purification System (Promega) as specified by the manufacturer. The sequencing reaction was performed using the ABI PRISM™ Dye Terminator Cycle Sequencing Ready Reaction Kit with Amplitaq DNA polymerase, FS as specified by the manufacturer. Sequencing products were analyzed using an ABI automatic sequencer model 377. Sense and antisense synthetic primers complementary to conserved eubacterial domains [44] were used to sequence both strands of the SSU rRNA gene. Accession numbers for these sequences are AJ785288 to AJ785292, and AJ785294.

### Sequence Analysis

The SSU rDNA sequences were compared to a database of aligned near full-length SSU rDNAs for each Rhizobiales species type strains [10] or the best sequence (longest and containing as few ambiguities as possible) for Rhizobiales lineages not represented by a type strain. The SSU-rDNA sequences for the rhizobial Australian genospecies that we had previously characterized [22] and the five sequences most similar to the sequences obtained in this study identified through Mega BLAST search (http://www.ncbi.nlm.nih.gov/BLAST/) were also included in the analyses.

The article "Molecular Diversity of Legume Root-Nodule Bacteria in Kakadu National Park, Northern Territory, Australia" was published in 2007. Journal: PLoS One.

Phylogenetic analyses were performed using near full-length aligned SSU rDNA sequences, only the extreme 5′-and 3′-ends of the alignment were excluded leaving 1472 sites, using PHYLIP 3.6b [45]. Trees were reconstructed by maximum likelihood using a gamma distribution with four rate categories and coefficients of variation (base frequencies, transition/transversion ratio, rates of change and gamma distribution shape parameter) estimated from the data using the DNAML programme. Statistical support for branching order was estimated from 100 bootstrap replications generated using SEQBOOT, using the CONSENSUS programme.
